# Dynamic Electrocardiogram under P Wave Detection Algorithm Combined with Low-Dose Betaloc in Diagnosis and Treatment of Patients with Arrhythmia after Hepatocarcinoma Resection

**DOI:** 10.1155/2021/6034180

**Published:** 2021-10-16

**Authors:** Fenfen Jiang, Haokai Xu, Xiaowen Shi, Bingjiang Han, Zhenliang Chu, Bin Xu, Xiaorong Liu

**Affiliations:** ^1^Department of Cardiology, The Second Affiliated Hospital of Jiaxing University, Jiaxing 314000, Zhejiang, China; ^2^Department of Surgery, Ningbo Yinzhou No. 2 Hospital, Ningbo 315199, Zhejiang, China; ^3^Department of Surgery, The Second Affiliated Hospital of Jiaxing University, Jiaxing 314000, Zhejiang, China

## Abstract

This work aimed to study the diagnostic value of dynamic electrocardiogram (ECG) based on P wave detection algorithm for arrhythmia after hepatectomy in patients with primary liver cancer, and to compare the therapeutic effect of different doses of Betaloc. P wave detection algorithm was introduced for ECG automatic detection and analysis, which can be used for early diagnosis of arrhythmia. Sixty patients with arrhythmia after hepatectomy for primary liver cancer were selected as the research objects. They were randomly divided into control group, SD group, MD group, and HD group, with 15 cases in each group. No Betaloc, low-dose (≤47.5 mg), medium-dose (47.5–95 mg), and high-dose (142.5–190 mg) Betaloc were used for treatment. As a result, P wave detection algorithms can mark P waves that may be submerged in strong interference. P waves from arrhythmia database were used to verify the performance of the proposed algorithm. The prediction precision (Pp) of ventricular arrhythmia and atrial arrhythmia was 98.53% and 98.76%, respectively. Systolic blood pressure (117.35 ± 7.33, 126.44 ± 9.38, and 116.02 ± 8.2) mmHg in SD group, MD group, and HD group was significantly lower than that in control group (140.3 ± 7.21) mmHg after two weeks of treatment. Moreover, those of SD group and HD group were significantly lower than MD group (*P* < 0.05). The effective rate of cardiac function improvement in SD group (72.35 ± 1.21%) was significantly higher than that in control group, MD group, and HD group (38.2 ± 0.98%, 65.12 ± 1.33%, and 60.43 ± 1.25%; *P* < 0.05). In short, dynamic ECG based on P wave detection algorithm had high diagnostic value for arrhythmia after hepatectomy in patients with primary liver cancer. It was safe and effective for patients to choose small dose of Betaloc.

## 1. Introduction

Liver cancer is a malignant tumor that occurs in the liver, the largest organ of the human body. It is generally classified into PHC and secondary liver cancer according to its etiology and other factors [1, 2]. PHC mainly includes hepatocellular carcinoma, intrahepatic cholangiocarcinoma, cholangiocarcinoma, angiosarcoma, hemangioendothelioma, and hepatoblastoma [3, 4]. At present, the preferred clinical treatment for liver cancer is hepatectomy, which is the traditional radical treatment for liver cancer, and the five-year survival rate of patients after surgery is greater than 50% [5, 6]. However, this surgery has certain limitations and is only suitable for patients with good liver function and complete tumor resection. In addition, it can lead to serious complications, such as liver failure and bleeding [7, 8]. Arrhythmia refers to when the origin of heartbeat excitement is abnormal or the conduction pathway is abnormal, and the sequence of excitement is disordered, which changes the heartbeat rate or rhythm [9, 10]. Arrhythmia is caused by a variety of triggers, and different clinical symptoms can occur due to different causes and types. In severe cases, syncope and sudden death can occur [11, 12]. In addition, a variety of treatments or antiarrhythmic drugs will have different degrees of side effects on patients. Therefore, when a drug is choosing for treatment, it is necessary to have a certain understanding of the pharmacokinetics and pharmacodynamics of the drug to prevent it from causing adverse reactions and complications to patients [13–15].

The ECG of arrhythmia shows that P wave appears in advance, and the shape is different from that of sinus P wave. PR interval is greater than 0.12 s. The QRS pattern is the same as that of sinus rhythm. In addition to accompanied by ventricle difference, conduction can appear inconsistent. There are usually incomplete compensatory intervals after pre-phase contraction of room type [16–18]. Detection of P wave is of great significance to ECG analysis of arrhythmia and analysis of characteristic points of ECG signal. Therefore, a P wave detection algorithm was proposed in this study to perform automatic detection and analysis of ECG and locate the P wave starting point, so as to achieve accurate and effective prediction and diagnosis of arrhythmia [19, 20]. At present, *β*-blocker drugs are gradually widely used in arrhythmia, especially in patients with primary liver cancer after hepatectomy, such as *β*-blocker metoprolol succinate sustained-release tablets (Betaloc) [21, 22]. However, because *β*-blockers have a certain blocking effect on *β*-receptors, there are certain limitations in clinical application [23, 24]. In addition, there is still a lack of relevant studies on the effect of dosage of *β*-blocker metoprolol succinate sustained-release tablets (Betaloc) on arrhythmia and its therapeutic effect [25, 26].

Therefore, in this study, patients with arrhythmia after hepatectomy for primary liver cancer were selected as the research objects, and no Betaloc, low-dose Betaloc, medium-dose Betaloc, and high-dose Betaloc were used for patients. By studying the cardiac function indexes, blood lipid indexes, and liver function indexes of different patients in different treatment periods, the therapeutic effect of low-dose Betaloc on arrhythmia after hepatectomy in patients with primary liver cancer was analyzed.

## 2. Materials and Methods

### 2.1. Basic Information

In this study, 60 patients with arrhythmia after hepatectomy for primary liver cancer who were hospitalized in hospital from September 2018 to October 2020 were selected as the research objects. Among them, 30 were male and 30 were female. They were randomly divided into control group, SD group, MD group, and HD group, with 15 cases in each group. No Betaloc, low-dose (≤47.5 mg), medium-dose (47.5–95 mg), and high-dose (142.5–190 mg) Betaloc were used for treatment. This study had been approved by the Ethics Committee of hospital, and patients and their families understood the study content and methods and agreed to sign corresponding informed consent forms.

Inclusion criteria were as follows: (i) patients aged between 40 and 65 years old; (ii) patients who were emotionally stable and can cooperate with treatment and sample collection; (iii) patients with arrhythmia after hepatectomy; (iv) patients with complete clinical data and information; (v) patients who had no history of mental illness and were emotionally stable; (vi) the left ventricular ejection fraction (LVEF) was less than 45%, and the left ventricular short axis fractional shortening (FS) was less than 25%; and (vii) patients with cardiac function grades III and IIII.

Exclusion criteria were as follows: (i) patients who withdrew and transferred for treatment due to personal reasons; (ii) patients with other serious diseases or infectious diseases; (iii) patients with diseases, such as hypertension and coronary heart disease, or similar surgical treatment experience; (iv) patients whose tumors had metastasized; and (v) patients who had not undergone cooperative treatment due to personal or other factors.

### 2.2. Required Sample Size Calculation

The required sample size is calculated as follows:

(1) $$\begin{array}{c} N=\frac{Z^{2}\times \left(P\times \left(1-P\right)\right)}{E^{2}}, \end{array}$$

(2) $$\begin{array}{c} n=\frac{Z^{2}\sigma^{2}}{d^{2}}. \end{array}$$

In equation (1), *N* is the total number of samples required in the experiment and *Z* is the statistic. When the confidence level is 95%, *Z* = 1.96. When the confidence is 90%, *Z* = 1.64%. *E* represents the error and *P* is the probability. In equation (2), *n* represents the required sample size for each group, *d* represents the sampling error range, and *σ* represents the standard deviation, which is generally 0.5. Through the above equations, it is calculated that *n* is 10, and the total number of samples required is 40 cases. In this study, 60 cases were selected, and there were 15 cases in each group.

### 2.3. ECG P Wave Detection Algorithm

The patient was placed in horizontal supine position with chest, wrist, and ankle exposed. The skin was cleaned with alcohol, and lead electrodes were placed to collect the electrocardiogram. Normal ECG signals are composed of P wave (from the point change of atrial depolarization before atrial contraction), QRS wave (from the change of ventricular depolarization before ventricular contraction), T wave (potential change during ventricular repolarization), PR segment, PR interval, ST segment, QT interval, and U wave with certain sequence (Figure 1).

The characteristic parameters related to P wave in ECG include P wave amplitude, PR interval, P wave duration, P wave dispersion, and atrial rate. P wave represents atrial depolarization, QRS wave represents ventricular depolarization, and T wave represents ventricular repolarization. In the actual ECG computer automatic analysis, the detected ECG signals are preprocessed first. The P wave amplitude is taken by the amplitude of the *P*-value. The PR interval refers to the beginning of the P wave to the beginning of the QRS wave, representing the time that the heart excited from the atria to the ventricles. The PR interval is divided into PA interval, AH interval, and HV interval, which is normally in the range of 120∼200 ms. PR interval is obtained according to the following equation:

(3) $$\begin{array}{c} \bar{PR}=\frac{\left(S_{Q}-S_{P}\right)}{t}. \end{array}$$

In equation (3), *S*_*Q*_ represents the starting point of QRS wave, *S*_*P*_ represents the starting point of P wave, and *t* represents the sampling rate. The P wave time limit refers to the process of left and right atrium depolarization and repolarization, with the general time (width) less than 0.12 s and the voltage (amplitude) less than 0.25 mV. In the analysis of electrical signals, the P wave time limit is calculated by the following equation:

(4) $$\begin{array}{c} \text{P wave duration}=\frac{\left(S_{P}-E_{P}\right)}{t}. \end{array}$$

In equation (4), *S*_*P*_ represents the starting point of P wave, *E*_*P*_ represents the end point of P wave, and *T* represents the sampling rate. P wave dispersion (PWD) refers to the difference between the maximum time (*Pm*) and the minimum time (*Pn*) measured in different leads of a 12-lead ECG recorded synchronically. The P wave dispersion of normal subjects is less than 40 ms, and the BBB 0 50 ms suggests the presence of heterogeneous electrical activity in different parts of the atrium P wave dispersion is a new index of body surface ECG in predicting atrial tachycardia and paroxysmal atrial fibrillation. The calculation method is shown in the following equation:

(5) $$\begin{array}{c} \text{P wave dispersion}=Pm-Pn. \end{array}$$

In equation (5), *Pm* represents the maximum time limit of P wave, and *Pn* represents the minimum time limit of P wave. The calculation method of heart rate is shown in the following equation:

(6) $$\begin{array}{c} \text{HR}=\frac{60\left(s\right)}{\bar{\text{PP}}or\bar{\text{RR}}\left(s\right)}. \end{array}$$

In equation (6), $\bar{\text{PP}}$ represents the average P-P interval and $\bar{\text{RR}}$ represents the average R-R interval.  Figure 2 shows the flow of P wave detection algorithm.

After the QRS is detected, the P wave search segment is determined, and the zero crossing between the mode extremum pairs in this segment is the P wave. The method to determine the mode extremum pair is shown in the following equations:

(7) $$\begin{array}{c} P_{x}=\frac{2}{5}\times \left(\frac{1}{10}\sum_{i=1}^{10}X_{i}\right), \end{array}$$

(8) $$\begin{array}{c} P_{y}=\frac{1}{3}\times \left(\frac{1}{10}\sum_{i=1}^{10}Y_{i}\right). \end{array}$$

In equations (7) and (8), *P* represents the amplitude, *X*_*i*_ represents the positive maximum value of the P wave search segment, and *Y*_*i*_ represents the negative maximum value of the P wave search segment. The local modulus maximum pairs are determined by screening the modulus extreme value pairs whose amplitude of point *A* was greater than *P*_*x*_ and that of point *B* less than *P*_*y*_, and the time interval was less than 100 ms. The detection of modulus extremum against slope is shown in the following equation:

(9) $$\begin{array}{c} K=\left|\frac{P_{A}-P_{B}}{P_{A}-P_{B}}\right|. \end{array}$$

In this study, the search criteria for P wave were as follows. The maximum value of the scale coefficient in the window was the modulus maximum point, the minimum value of the scale coefficient was the modulus minimum point, and the zero crossing between them was the P wave.

### 2.4. Drug Therapy for Patients

The patients in the control group, SD group, MD group, and HD group were guided and managed in the course of medication and diet after surgery. In addition, the real-time monitoring was performed on the heart and lung function indexes, blood gas analysis indexes, and psychological status of each group of patients. The four groups of patients were treated with different doses of beta-blocker metoprolol succinate sustained-release tablets (Betaloc) after surgery.

No Betaloc was adopted by patients in control group. SD group: initial dose of Betaloc was 12 to 24 mg once a day, and the patient's tolerance was observed the next day. If the patient could tolerate the previous daily dose, the dose was doubled three weeks later and increased to the target dose of 47.5 mg in SD group. If the patient had adverse reactions or drug intolerance, it was necessary to reduce the drug dose and stop using it in severe cases. In addition, other agents were used or the Betaloc dosage was gradually restored after the patient's condition became stable. MD group: the initial dose of Betaloc was 12 to 24 mg once a day, and the patient tolerance was observed the next day. If the patient could tolerate the previous daily dose, the dose was doubled three weeks later and increased to the target dose of 47.5–95 mg in the MD group. If the patient had adverse reactions or drug intolerance, it was necessary to reduce the drug dose and stop using it in severe cases. In addition, other agents were used or Betaloc dosage was gradually restored after the patient's condition became stable. In the HD group, the initial dose of Betaloc was 12 to 24 mg once a day, and the patient's tolerance was observed the next day. If the patient could tolerate the previous daily dose, the dose was doubled three weeks later, and the target dose was successively increased to 142.5–190 mg as that of the HD group. In the case of adverse reactions or drug intolerance in patients, the drug dose should be reduced and discontinued in severe cases, and the dosage of Betaloc should be gradually resumed after the patient's condition became stable.

### 2.5. Evaluation Indexes

The four groups of patients were treated with different treatment methods and doses. In addition, the patients' heart function indexes, blood lipid indexes, liver function indexes, and ECG signal were detected before and at different periods after treatment, including diastolic blood pressure, systolic blood pressure, heart rate, B-type natriuretic peptide precursor (pre-proBNP), blood sugar (GLU), cholesterol (TC), triglycerides (TG), alanine aminotransferase (ALT), aspartate aminotransferase (AST), and types and incidence of complications.

### 2.6. Statistical Methods

SPSS 19.0 was employed for data statistics and analysis. Mean ± standard deviation ($\bar{x}\pm s$) was how measurement data were expressed, and percentage (%) was how count data were expressed. Pairwise comparison adopted analysis of variance. The difference was statistically considerable with *P* < 0.05.

## 3. Results

### 3.1. ECG Signal Monitoring in Patients with Arrhythmia

Figure 3 shows the ECG signal monitoring record of patients with arrhythmia. In Figure 3(a), there was no relationship between the central atrial wave and the ventricular wave, showing a complete disconnection. The atrial rate was 88 bpm, the ventricular rate was 30 bpm, the atrial rate was greater than the ventricular rate, and the Q-T interval was 0.68 s. In Figure 3(b), the P wave appeared regularly, with a frequency of 62 bpm. After the first, third, and fourth P waves, there were downstream QRS-T complexes. QRS-T complexes without downcoming after the 5th wave were type I atrioventricular block.

Figure 4 shows the detection results of ECG signal. It was found that the P wave detection algorithm can mark the P wave, which may be submerged in strong interference, accurately locate the P wave and T wave peaks of ECG signal, and detect the P wave and T wave singularity. The diagnostic error rate (Er), sensitivity (Se), and prediction precision (Pp) of P wave detection algorithm for ventricular arrhythmia were 0.24%, 99.23%, and 98.53%, respectively. Er, Se, and Pp of atrial arrhythmia were 0.28%, 99.45%, and 98.76%, respectively.

### 3.2. Basic Patient Information

Figure 5 shows the comparison results of the basic information of the four groups of patients before treatment.  Figure 5(c) shows the number of patients with cardiac function grades of grade III and IIII.  Figure 5(d) shows the number of patients with mild heart failure, moderate heart failure, and no heart failure. There was no considerable difference in the proportion of patients with different ages, genders, heart function grades, and combined heart failure in each group (*P* > 0.05).

### 3.3. Changes of Diastolic Blood Pressure, Systolic Blood Pressure, and Heart Rate before and after Treatment

Figure 6(a) shows the changes in systolic blood pressure of the four groups of patients before treatment, one week after treatment, and two weeks after treatment. With the treatment time, the systolic blood pressure of the four groups of patients gradually decreased. After one week of treatment, patients in the SD group and HD group had lower systolic blood pressure, while the control group had higher systolic blood pressure. The systolic blood pressure of the SD group, MD group, and HD group after two weeks of treatment (117.35 ± 7.33 mmHg, 126.44 ± 9.38 mmHg, and 116.02 ± 8.2 mmHg) were significantly lower versus that of control group (140.3 ± 7.21 mmHg), and that of SD group and HD group was greatly inferior to the MD group (*P* < 0.05).  Figure 6(b) shows the changes in diastolic blood pressure of the four groups of patients before treatment, one week after treatment, and two weeks after treatment. The diastolic blood pressure of the SD group was considerably inferior to that of the control group one week after treatment (*P* < 0.05). After two weeks of treatment, the diastolic blood pressure (74.12 ± 9.38 mmHg, 88.15 ± 8.2 mmHg, and 84.33 ± 7.21 mmHg) of the SD group, MD group, and HD group was substantially lower relative to that of control group (95.38 ± 7.33 mmHg), and that of SD group was evidently lower versus that of MD group and HD group (*P* < 0.05).  Figure 6(c) shows the heart rate changes of the four groups of patients before treatment, one week after treatment, and two weeks after treatment. The heart rate of the SD group after two weeks of treatment was obviously inferior to that of the control group and the HD group (*P* < 0.05).  Figure 6(d) shows the comparison results of the pre-proBNP content of type B natriuretic peptide of the four groups of patients. The pre-proBNP of SD group was notably lower versus that of control group, MD group, and HD group, and MD group was lower than HD group (*P* < 0.05).

### 3.4. Comparison on the Effective Rate of the Improvement of the Heart Function

Figure 7 shows the comparison results of the changes in the effective rate of cardiac function improvement after the four groups of patients were treated with different doses of Betaloc for 1, 2, and 3 weeks. After one week of treatment, patients in the MD and HD groups had a relatively higher effective rate of improvement in heart function. With the treatment time, the effective rate of cardiac function improvement of the four groups of patients gradually increased. After three weeks of treatment, the effective rate of cardiac function improvement (72.35 ± 1.21%) in the SD group was notably superior to that of the control, MD, and HD groups (38.2 ± 0.98%, 65.12 ± 1.33%, and 60.43 ± 1.25%) (*P* < 0.05).

### 3.5. Analysis of Blood Lipid Indexes before and after Treatment

Figure 8(a) shows the comparison results of the GLU content of the four groups of patients before and after treatment. There was no remarkable difference in the GLU content among the control group, SD group, MD group, and HD group before treatment (*P* > 0.05). After treatment, the GLU content of the SD group (5.84 ± 0.62 mmol/L) was greatly higher than that of the control group, MD group, and HD group (4.56 ± 0.58 mmol/L, 4.97 ± 0.49 mmol/L, and 5.09 ± 0.54 mmol/L) (*P* < 0.05). Figures 8(b) and 8(c) present the comparison results of the TC content and TG content of the four groups of patients before and after treatment, respectively. There was no considerable difference in TC content and TG content among the control group, SD group, MD group, and HD group before treatment (*P* > 0.05). After treatment, the TC content and TG content of the SD group were dramatically superior to those of the control group, MD group, and HD group (*P* < 0.05).

Figure 9 shows the comparison results of the changes in liver function indexes ALT and AST content of the four groups of patients. From Figure 9(a), there was no substantial difference in ALT content among the four groups of patients after one week of treatment (*P* > 0.05). After two weeks and three weeks of treatment, the ALT content of the SD group was remarkably inferior to that of the control group, MD group, and HD group, and that of MD group and HD group was greatly lower versus control group (*P* < 0.05). From Figure 9(b), the AST content of the SD group and the HD group was notably lower than that of the control group and the MD group after two weeks of treatment, and that of MD group was dramatically lower relative to control group (*P* < 0.05). After three weeks of treatment, the content of SD group was substantially lower than that of control group, MD group, and HD group (*P* < 0.05).

### 3.6. Complications in the Four Groups

Figure 10 shows the types and incidence of complications in the four groups of patients before and during treatment. From Figures 10(a) and 10(b), patients with PHC undergoing hepatectomy for arrhythmia were prone to hypertension, diabetes, atrial fibrillation, postoperative arrhythmia, atrioventricular block, sinus bradycardia, hypotension, nausea and vomiting, headache, dizziness, etc. From Figure 10(c), the incidence of the above complications in the control group, SD group, MD group, and HD group was 34.6%, 12.4%, 20.5%, and 32.5%, respectively. The incidence of the above complications was the lowest in the SD group, followed by the MD group and the HD group.

## 4. Discussion

ECG records at the onset of arrhythmias are important evidence for the diagnosis of arrhythmias. During diagnosis, emphasis should be placed on checking whether the patient has organic heart disease such as hypertension, coronary heart disease, and myocarditis, and some physiological and pathological factors can cause arrhythmias [27, 28]. Physiological factors include exercise and emotional excitement, while pathological factors include cardiovascular diseases and endocrine diseases [29, 30]. Studies found that Betaloc is the drug with the lowest side effects among all drugs for the treatment of arrhythmia, and the only drug that can reduce the mortality rate of the disease. It can not only be applied to angina pectoris and myocardial infarction, but also can effectively reduce myocardial oxygen consumption, slows heart rate, reduces angina pectoris, and effectively prevents arrhythmia after myocardial infarction [31–33]. Kotecha et al. [34] found that due to differences in physique and drug response of different patients, whether it is angina pectoris, arrhythmia, or heart failure, if Betaloc is selected as a therapeutic drug, it is necessary to start taking a small dose. If adverse reactions such as drug intolerance occur, it is necessary to stop taking it. The study of Blessberger et al. [35] found that Betaloc, as a beta-blocker, can slow down heart rate, reduce myocardial contractility, and thereby lower blood pressure. It mainly acts on the heart and has certain effects on bronchial smooth muscle. Although drugs such as Betaloc can reduce the heart rate and protect the heart, if the condition is unstable (when the condition is severe or acute left heart failure) for patients with arrhythmia or heart failure, they should avoid taking such drugs without authorization [36]. When heart failure worsens, fast heart rate is also a kind of self-protection. It is necessary to control the heart failure to a stable state before using Betaloc to lower the heart rate. Forcibly suppressing the heart rate when heart failure worsens will have a greater impact on the patient, and even life-threatening [37–39].

The P wave detection algorithm was introduced to detect and analyze the ECG automatically, and it was used in the early diagnosis of arrhythmia. Patients with arrhythmias after hepatectomy for PHC were selected as subjects and treated with different doses of Betaloc. The cardiac function indexes, blood lipid indexes, and liver function indexes of patients at different stages of treatment were analyzed; the therapeutic effect of low-dose Betaloc on arrhythmia after hepatectomy in patients with PHC was analyzed. As a result, the P wave detection algorithm can accurately locate the P wave and T wave peaks of the ECG signal. The diagnostic error rate, sensitivity, and correct prediction of ventricular arrhythmia were 0.24%, 99.23%, and 98.53%, respectively. The diagnostic error rate, sensitivity, and correct prediction of atrial arrhythmia were 0.28%, 99.45%, and 98.76%, respectively. Therefore, the proposed P wave detection algorithm had high application value for the diagnosis and early prediction of arrhythmia. The heart rate of the SD group after two weeks of treatment was obviously lower versus control group and the HD group (*P* < 0.05), which suggested that Betaloc can reduce the heart rate of patients with arrhythmia, and the effect of low-dose Betaloc in reducing the heart rate was the most obvious. The effective rate of cardiac function improvement in SD group (72.35 ± 1.21 mmHg) was remarkably superior to that of control group, MD group, and HD group (38.2 ± 0.98 mmHg, 65.12 ± 1.33 mmHg, and 60.43 ± 1.25 mmHg) (*P* < 0.05), which suggested that a small dose of Betaloc can significantly improve the cardiac function of patients with arrhythmia. After two weeks and three weeks of treatment, the ALT content of the SD group was substantially inferior to that of the control group, MD group, and HD group, and that of MD group and HD group was greatly lower versus control group (*P* < 0.05). After two weeks of treatment, the AST content of the SD group and the HD group was considerably lower versus control group and the MD group, and that of MD group was notably lower versus control group (*P* < 0.05). After three weeks of treatment, the content of SD group was evidently lower than that of control group, MD group, and HD group (*P* < 0.05), which was consistent with the results of Irizarry-Alvarado [40], indicating that patients with arrhythmia after PHC hepatectomy were safer to choose low-dose Betaloc, which had a good curative effect, can effectively reduce the heart rate, reduced the occurrence of complications, and improved heart function.

## 5. Conclusion

In this study, the automatic detection and analysis of ECG was carried out by introducing the P wave detection algorithm, and it was used for the early diagnosis of arrhythmia. Different doses of Betaloc were used to treat arrhythmia, so as to study the therapeutic effect of low-dose Betaloc on the complications of arrhythmia after hepatectomy in patients with primary liver cancer. The results suggested that dynamic ECG based on P wave detection algorithm had high diagnostic value for arrhythmia after hepatectomy in patients with primary liver cancer. The low-dose Betaloc used by patients was safer and had relatively better curative effect. However, the sample size selected in this study is small, which may have a certain impact on the experimental results, and the representativeness is low. Therefore, in the follow-up experiments, the sample size will be increased, and the application of Holter based on P wave detection algorithm combined with low-dose Betaloc in the diagnosis and treatment of arrhythmia after liver cancer resection will be further studied.

## Figures and Tables

**Figure 1:** Waveform diagram of ECG signal.

**Figure 2:** ECG detection process (a) and P wave detection process (b).

**Figure 3:** Patient's ECG signal monitoring chart. (a) ECG signal monitoring chart of a patient with arrhythmia. (b) ECG signal monitoring chart of patient with arrhythmia combined with atrioventricular block.

**Figure 4:** ECG signal detection results. (a) P and T wave detection results (P means P wave and T means T wave). (b) Arrhythmia diagnosis results.

**Figure 5:** Comparison of the basic information of the four groups of patients. (a) Age. (b) Gender ratio. (c) Heart function level before treatment. (d) Patients complicated with heart failure.

**Figure 6:** Changes of cardiac function indexes in the four groups. (a) Systolic blood pressure; (b) diastolic blood pressure; (c) changes in heart rate; (d) the pre-proBNP. ^*∗*^ represents significant difference compared with control group (*P* < 0.05); # represents significant difference compared with HD group (*P* < 0.05); Δ represents significant difference compared with MD group (*P* < 0.05).

**Figure 7:** Comparison of the effective rate of cardiac function improvement in the four groups of patients. ^*∗*^ indicates considerable differences versus control group (*P* < 0.05); # indicates considerable differences versus HD group (*P* < 0.05); Δ indicates considerable differences versus MD group (*P* < 0.05).

**Figure 8:** Comparison of blood lipid indexes of the four groups of patients before and after treatment. (a) GLU comparison before and after treatment. (b) TC comparison. (c) TG comparison. ^*∗*^ indicates considerable differences versus control group (*P* < 0.05); # indicates considerable differences versus HD group (*P* < 0.05); and Δ indicates considerable differences versus MD group (*P* < 0.05).

**Figure 9:** Analysis of liver function indexes of four groups of patients. (a) Changes in ALT content. (b) Changes in AST content. ^*∗*^ represents remarkable versus control group (*P* < 0.05).

**Figure 10:** Complications occurred in the four groups of patients. (a, b) The types of complications in the four groups of patients. (a, b, c, d, e, f, g, h, and i indicate hypertension, diabetes, atrial fibrillation, atrioventricular block, sinus bradycardia, hypotension, nausea and vomiting, headache, and dizziness, respectively). (c) The complication rate.

## Data Availability

The data used to support the findings of this study are available from the corresponding author upon request.
